# Comparison of Extracorporeal Shock Wave Therapy versus Manual Lymphatic Drainage on Cellulite after Liposuction: A Randomized Clinical Trial

**DOI:** 10.1155/2021/9956879

**Published:** 2021-08-10

**Authors:** Nesma M. Allam, Radwa T. Elshorbagy, Marwa M. Eid, Walid Kamal Abdelbasset, Safaa Mostafa Elkholi, Hadaya Mosaad Eladl

**Affiliations:** ^**1**^ Department of Physical Therapy for Surgery, Faculty of Physical Therapy, Cairo University, Giza, Egypt; ^**2**^ Department of Physical Therapy, College of Applied Medical Sciences, Jouf University, Sakaka, Saudi Arabia; ^3^Department of Physical Therapy for Musculoskeletal Disorders & Its Surgery, Faculty of Physical Therapy, Cairo University, Giza, Egypt; ^4^Department of Physical Therapy, College of Applied Medical Sciences, Taif University, Taif, Saudi Arabia; ^5^Department of Health and Rehabilitation Sciences, College of Applied Medical Sciences, Prince Sattam Bin Abdulaziz University, Al Kharj, Saudi Arabia; ^6^Department of Physical Therapy, Kasr Al-Aini Hospital, Cairo University, Giza, Egypt; ^7^Department of Rehabilitation Sciences, Faculty of Health and Rehabilitation Sciences, Princess Nourah Bint Abdulrahman University, Riyadh, Saudi Arabia

## Abstract

**Introduction:**

Cellulite is associated with variations in the skin appearance with cottage cheese, mattress-like, or orange peel. The most common areas for these lesions are the posterior or upper thighs and buttocks and mainly affect females after puberty. The objective of the study was to determine whether extracorporeal shock wave therapy (ESWT) or manual lymphatic drainage (MLD) is more effective for the reduction of the grade of cellulite after liposuction.

**Methods:**

This study is a single-blinded randomized controlled clinical trial. Thirty females with grade 3 cellulite were randomly distributed into two groups equal in number (*n* = 15), group A was equipped to ESWT and group B was equipped to MLD. The cellulite grading scale was used to assess cellulite grade, and the skinfold caliper was used to assess the thickness of subcutaneous fat. The assessment was carried out before and four weeks after starting the treatment. Both groups received topical retinol twice daily for four weeks; in addition, group A received ESWT, while group B received MLD, two times/week for 4 weeks.

**Results:**

The mean values of the skinfold caliper in group A decreased by 24.4% and in group B by 15.38% with a significant difference between the two groups (*p* < 0.001). Also, the mean values of the cellulite grading scale decreased significantly after treatment in group A compared with the mean values of group B (*p* < 0.001).

**Conclusions:**

There was more reduction in the grade of cellulite and thickness of subcutaneous fat in the ESWT group than the MLD group after liposuction.

## 1. Introduction

Cellulite is a common disorder affecting the subcutaneous tissue associated with changes of the skin topography due to structural and biochemical components. It appears as depressions and bulges that present mainly in the lower limbs and the gluteus area [1–3].

The most frequent risk factors contributing to cellulite formation are hormonal factors, genetic predisposition, inadequate diets, inactivity, excess body fat, smoking, postural disorders, and wearing tight clothes that cause external compression on body parts. The incidence of cellulite is about 85%–98% in women [4].

The deposition of excess fat may affect the hormonal function that eliminates the lipolytic enzymes' levels. Fat cells are located between the superficial layer of the dermis and underlying muscle fibers in the fibrillary network [5]. Cellulite occurs due to the elimination of stimulation of the venous and lymphatic vessels, which reduces the lymphatic drainage. Therefore, accumulation of fluid occurs within the dermis and subcutaneous tissues [6].

The most common method used to classify cellulite is the cellulite grading scale that was classified into four grades defined by clinical manifestation: grade zero: no differences; grade I: noticeable differences at the pinch test; grade II: noticeable differences associated with manipulation; and grade III: noticeable differences during nodulations [7].

Liposuction surgery is defined as a surgical procedure applied to remove fat from subcutaneous tissues by using metal cannulas that are placed through small incisions. Liposuction can secondarily worsen the degree of cellulite by reducing the amount of subcutaneous fat [8].

Liposuction most commonly causes changes in the cutaneous surface, which have the same appearance as the skin depression of cellulite. These depressed lesions cause secondary cellulite or exacerbate the grade of cellulite [9].

Shock waves are focused high-pressure acoustical waves characterized by a very short time of application (<1 microsecond) with a pressure of 10–100 MPa and a low-wave component (10% of maximum pressure). They are transmitted without major losses through soft tissue [10].

Shock wave was used to remove stones within the body. ESWT has now been chosen for the treatment of renal calculi. ESWT was most commonly used as an effective modality for most musculoskeletal deficits. Shock wave therapy is a new modality for the improvement of cellulite and lipedema; it is an easy, noninvasive, local therapy, without side effects, with short periods of application. Its original idea was the stimulation of lipid mobilization and improved lipolysis in areas with edema [11].

High-focused ESWT with medium energy was applied to the skin as a noninvasive therapy approach for cellulite. Recently, treatment with low-energy unfocused ESWT has shown evidence of collagen remodeling in the dermis. In addition, application of laser or radiofrequency (RF) was beneficial for the improvement of the grade of cellulite [12].

Manual lymphatic drainage is a technique performed for stimulation of the lymphatic system, decrease of extra fluid, and reduction of the metabolic waste, and as cellulite is related to the accumulation of fluid in the dermis and metabolic changes causing disturbances in anatomical structures, MLD may be effective in improving the cellulite appearance [13].

The purpose of MLD is to drain the accumulated fluids between interstitial spaces, especially in the dermis, for maintaining the balance of the tissue fluid by differences of pressure that will enhance the transport of lymph fluid into the blood vessels by application of superficial and deep techniques along the pathway of the lymphatic system [14].

Prior researches focused on the impact of ESWT [15–17] and MLD [6, 13] on cellulite. To the best of our knowledge, studies of comparison between the effect of ESWT and MLD on cellulite following liposuction are limited. The current study, therefore, aims to detect which is more effective, the extracorporeal shock waves therapy or manual lymphatic drainage, in the elimination of cellulite grade after liposuction.

## 2. Methods

### 2.1. Study Design

This is a single-blinded randomized clinical trial. It was ethically approved by the Faculty of Physical Therapy ethical committee, Cairo University, Giza, Egypt (No: P.T.REC/012/002757), and registered by ClinicalTrials.gov with identifier, NCT04498312. Participants were informed about the nature, purposes, and benefits of the study in detail. Each participant signed informed consent before participation in the study.

### 2.2. Subjects

Thirty participants were enrolled randomly to participate in this study from the Plastic Surgery Department, Kasr Al-Aini Hospitals. Group A (ESWT group) (*n* = 15) received extracorporeal shock wave therapy twice/week for four weeks plus topical retinol twice daily for 4 weeks; group B (MLD group) (*n* = 15) received manual lymphatic drainage twice a week for four weeks plus topical retinol twice daily for 4 weeks.

Participants were selected according to the following criteria: Female patients with age ranged from 25–45 years, nonpregnant females, and grade 3 cellulite following liposuction at the thigh level. The exclusion criteria included the following: breastfeeding females, inflammatory skin disorders in the treatment area, edema, varicose veins, any therapy that may affect treatment (received chemotherapy, anticoagulation therapy, and cortisone therapy), morbid obesity (BMI >40), and diseases that may affect treatment (cardiac disease, hepatic disease, hyperthyroidism, thrombosis, malignoma, diabetes mellitus, or hypercholesterinemia). Participants were asked not to attend any exercise or diet programs that would change their weight.

### 2.3. Randomization

Forty-five patients underwent eligibility tests within the Outpatient Clinic of the Faculty of Physical Therapy, Cairo University. Randomization was conducted by using sealed envelopes that were randomly filled from a bowl with cards filled with either ESWT or MLD. Participants were blinded during allocation. Randomization was carried out by a blinded investigator. The participants were distributed to their groups according to the selected card. The data collection was conducted at baseline and after the end of the intervention period.

### 2.4. Sample Size Calculation

For sample size calculation, the G ^*∗*^ power 3.1 software (Universities, Düsseldorf, Germany) was utilized. The sample size was computed based of the cellulite grading scale, which is the primary outcome of the current study with 80% power, *α* = 0.05, *β* = 0.2, effect size = 0.4, and revealed that 12 participants are the required sample size for each group.

### 2.5. Outcome Measures

The primary outcome measure was the cellulite grade, and the secondary outcome measure was the thickness of subcutaneous fat. Both were measured at baseline and after 4 weeks of treatment.

The cellulite grading scale was used for assessment of cellulite grade score by inspection while the patient was in the standing or lying position. Grade (0) means a smooth skin surface when the patient is standing, grade (1) means pinch-test mattress phenomena, grade (2) means phenomena of the mattress spontaneously when standing, and grade (3) means phenomena of the mattress while standing and lying [7].

The thickness of subcutaneous fat was assessed using a skinfold digital caliper (SKYNDEX System I, Caldwell, Justiss and Company, Inc. Fayetteville, AR, USA). Measurements were taken at the thigh area to detect the thickness of the subcutaneous fat. The measurement procedure was conducted at the same time as the date while the patient is in a standing position. These measurements were taken from the midpoint of the line that crosses the center of the patella point and the anterior upper iliac spine. The caliper was at a right angle with the skin; the measurement was performed on the skin and subcutaneous fatty tissues, not the muscles, as the thickness of the muscles made the thickness denser [18]. A skinfold was lifted between the thumb and forefinger for the area to be measured, and the calipers were applied 1-2 cm away and approximately in the middle of the fold. After the calipers were applied, the needle movement often continued, and the reading was taken after all movements had ceased. The author, who was responsible for the assessment, took three readings of skinfolds in different directions at the same site [6]. After waiting two seconds with the calipers engaged, the measurement was taken. Then, the calipers were released, and another measurement was taken. For each subject, three measurements were averaged [19].

### 2.6. Intervention

#### 2.6.1. Extracorporeal Shock Wave Therapy Procedure

ESWT (STORZ Medical AG, Switzerland) with radial waves (D-Actor applicator) was used with the following parameters: (0.1–8.0 energy level, 3.5 mean energy level, and 0.16 mJ/mm^2^ energy flux density) for each thigh. The patient was in a supine lying position with the areas to be handled exposed when the shock wave head was applied to the anterior portion of the thigh that was scanned for both horizontal and vertical directions with 2000 shots 2 times/week for 4 weeks [12, 15].

#### 2.6.2. Manual Lymphatic Drainage Procedure

It was introduced by applying pressure manually toward the direction of the lymphatic system. The pressure was applied by sliding the hands through the pathway of the lymphatic system up to the related lymph nodes. First, the abdominal region was treated with MLD from the supine lying position, and the inguinal lymph nodes were subsequently stimulated. The participant then turned to a prone lying position; MLD started from above the tendoachilis area to the popliteal lymph nodes. Again, the popliteal lymph nodes were stimulated once more after the thigh was drained. Then, the thigh area again drained up toward the inguinal lymph nodes, in a circular manner by the hand wrapping around the thigh circumferentially from all directions getting the lymphatic drainage in upward direction. The lymphatic drainage of the thigh and the lymph nodes was next stimulated again. The period of the session was 60 minutes ^13^, and it was applied twice/week for four weeks [6, 14, 20].

### 2.7. Topical Retinol

A stabilized retinol formulation (Retinol ActifPur®, Roche) was applied twice daily for 4 weeks on the affected area for both groups [21]. The amount to be applied was demonstrated by creating a layer of about 0.1 mm to coat the affected area, and gentle massage was applied for equal distribution of the topical treatment on the whole area [22].

### 2.8. Statistical Analysis

A comparison of characteristics of subjects between both groups was conducted by descriptive statistics and unpaired *t*-test. For normal data distribution, the Shapiro–Wilk test was used. Levene's test for variances homogeneity was carried out to assess the homogeneity between groups. A comparison of the values of the skinfold caliper between groups A and B was carried out by the unpaired *t*-test. A paired *t*-test was carried out for comparison of the skinfold caliper between pretreatment and after four weeks in each group. The cellulite grading scale was compared between groups by the Mann–Whitney *U* test and compared between pretreatment and four weeks after treatment in each group by Wilcoxon Signed Ranks. The significance level was *p* < 0.05 for the statistical tests. The SPSS was used with windows (V. 22, IBM SPSS, Armonk, NY, USA) for all statistical analysis.

## 3. Results

Forty-five female participants were selected for eligibility. Fifteen participants were excluded (8 did not match the inclusion criteria of the study, and 7 declined to participate in the study). Thirty participants were assigned randomly into two groups of 15 participants per group. All participants were assessed before treatment and after four weeks and received the treatment procedures without withdrawal, as shown in the flow chart in Figure 1.

Table 1 shows the characteristics of subjects of the group A (ESWT group) and B (MLD group). No statistically significant difference was noted between both groups in the mean values of age, height, and weight in addition to BMI (*p* > 0.05).

Mean values of the skinfold caliper were significantly decreased in after treatment in both groups compared with that before treatment (*p* > 0.001). The percent of the decrease in the skinfold caliper in groups A (ESWT group) and B (MLD group) were 24.4 and 15.38%, respectively, as shown in Table 2. A significant improvement was recorded in the cellulite grading scale after treatment in both groups compared with that before treatment (*p* < 0.001), as presented in Table 3.

No significant difference was recorded in the skinfold caliper and cellulite grading scale between groups before treatment (*p* > 0.05). A significant decrease in the skinfold caliper and cellulite grading scale was recorded in group A (ESWT group) compared with group B (MLD group) after treatment (*p* < 0.001), as displayed in Tables 2 and 3 and Figures 2 and 3.

There were no side effects for both interventions except slight redness immediately after the session which disappears within 24 hours after the session.

## 4. Discussion

This study compared the effect of ESWT versus MLD on 30 females with grade 3 cellulite, and a significant decrease in the skinfold caliper and cellulite grading scale was recorded in group A compared with group B (*p* < 0.001) after comparison between both groups after treatment. The percent of the decrease in the skinfold caliper in the ESWT group and MLD group was 24.4 and 15.38%, respectively.

Cellulite can appear in any area of the body that contains subcutaneous fat. Cellulite most commonly affects women more than men. It mainly occurs in the abdomen, buttocks, pelvic region, and thighs. Cellulite mainly causes changes in the skin without changes in fat cells. Although cellulite often affects healthy normal-weighted patients, obesity can trigger its composition. In some patients, loss of weight may worsen the grade of cellulite [21, 22].

Cellulite results from decreased transport capability of the lymphatic system. At lipedema (advanced stage of cellulite), there is an inability of the lymphatic vascular system to transfer an adequate quantity of protein molecules from the interstitium to the venous bloodstream. As a result, the concentration of plasma proteins present in the interstitium increases, which produces fibrosis and, thus, changes the tissue properties [23, 24]. One of the topical treatments used to treat cellulite is retinoids that proved to reduce the degree of cellulite by increasing the thickness of the dermis, angiogenesis, formation of new connective tissue structures, and enhancing the number of fibroblasts [22].

There is evidence at radial and focused ESWT, and their combination improves the cellulite grade and skin appearance and decreases the thickness of the subcutaneous fat. It was proved that 6–8 sessions once or twice/week have been effective in most studies. There is a lack of combination therapies with other modalities such as as cryolipolysis, low-level laser, or others [25].

Russe-Wilflingseder et al. assessed the efficacy of ESWT on 11 women with cellulite. Six sessions were applied with radial ESW D-Actor (3 bars, 10 Hz, and 2000 impulses) on the upper leg and buttock every 7 days. The results proved that radial ESWT is effective and safe for cellulite treatment with no side effects [16]. In addition, Christ et al. designed a study on 69 women with grade 2-3 cellulite and evaluated the effect of ESWT on skin elasticity for 6 sessions. They concluded that acoustic wave therapy improves the grade of cellulite by improving the microcirculation and transport capability of lymph vessels [17]. Adatto et al. evaluated the effect of radial ESWT on 25 women. They applied 6 sessions with ESWT D-Actor (2.6–3.6 bar, 15 Hz, and 3000 impulses) twice per week with follow-up at 12 weeks. All patients were assessed by using the Derma Lab Device for skin elasticity. The results proved that skin elasticity was improved after the first follow-up visit [1].

Also, Angehrn et al. investigated the effect of shockwave on cellulite. They performed the study on 21 women who received 12 sessions of unfocused ESWT over 6 weeks in the lateral thigh [11]. They reported an increase in the skin elasticity, measured by ultrasound of high resolution and a self-assessment questionnaire. Furthermore, Knobloch et al. evaluated the efficacy of ESWT with exercise in cellulite treatment. Focused ESWT (0.35 mJ/mm^2^, 2000 impulses) was applied on the gluteal and thigh areas for 6 sessions every 1 to 2 weeks for the study group. Sham-ESWT was applied to participants in the control group [26]. Both groups received gluteal strength exercises daily. The cellulite grade and the skin appearance were significantly improved, but it was ineffective on decreasing thigh circumference.

Also, Siems et al. investigated the effectiveness of ESWT in cellulite and found that acoustic waves cause disruption of the sclerotic fibrous septae that causes the cellulite appearance. In addition, acoustic wave therapy caused a decrease in fat thickness [27].

Furthermore, other studies concluded that ESWT was the preferable modality for cellulite treatment with the improvement of elasticity and appearance of the skin. It was proved that microcirculation and lymph flow was also boosted. In addition, lipolysis was increased by acoustic waves, which tightened skin and achieved a significant reduction of the treated area [28–33].

Stimulation of the drainage of the lymph fluid is the basis of cellulite treatment. This technique included cervical stimulation and mechanical and manual lymphatic drainage, which stimulate contraction and mobility of lymphatic vessels [34, 35].

The MLD technique is a procedure in which the blocked lymphatic fluid can circulate freely by manual manipulation of the lymphatic system. This strengthens the adipose tissue, reduces the intercellular edema of the fat tissue, increases the lymphatic flow, and speeds up the drainage of the lymphatic fluid into lymphatic channels. The effects on the sympathetic nervous system relieve pain and provide a deep sense of comfort. This supports immunity. MLD encourages the synthesis of collagen in the skin and so tightens the skin [6].

In addition, Adriana et al. performed a study on ten women with cellulite and investigated the effectiveness of MLD with ultrasound (US) for treating cellulite. MLD was applied for 60 minutes, and the US was applied on the upper thigh and the buttocks for 12 minutes. The results showed that cellulite and the patient's satisfaction were significantly improved [36].

Furthermore, Godoy and Godoy conducted a study on 14 patients who participated in the treatment program for cellulite for 10 sessions over 2 weeks by cervical stimulation and manual and mechanical lymphatic drainage. Results showed that lymphatic drainage was effective for the treatment of cellulite. This drainage technique is dependent on hydrodynamic, anatomy, physiology, and pathophysiology principles for fluid drainage in lymphatic collectors [37].

Also, Bayrakci et al. investigated the effect of manual lymphatic drainage, manipulation of connective tissue, and mechanical massage on fat thickness and cellulite. Their study was carried out on 60 participants. Results showed a decrease in the thickness of fat tissues after the treatment. Also, there was an improvement in cellulite [6].

The explanation that ESWT has a positive effect on cellulite reduction better than MLD may be referred to as its stronger effect on collagen remolding. Shockwave energy might have weakened the fibrous septae, and thus, the afflicted skin became smoother.

In accordance with the findings of the current study, Schonvvetter et al. proved that MLD was ineffective when performed in isolation to change the dermis, dermal hypodermal interface, although it was effective in the reduction of the hip circumference, with a positive effect on the quality of life [38]. On the contrary, Goody et al. proved that manual lymphatic drainage was effective for the treatment of cellulite; treatment was based on manual lymph drainage with one session per day for 10 days using the technique developed in [39]. This technique is characterized by movements that compress and subsequently slide along the route of the lymphatic vessels, the great saphenous lymphatic chain, up to the corresponding lymph nodes, fifteen minutes per day of cervical stimulation.

This study has the following drawbacks: small sample size and the number of sessions for ESWT and MLD; another limitation was the lack of the follow-up period due to limited time and funding. Additional studies are needed to investigate a higher number of patients, apply treatment procedures for longer periods, with some sort of control group that receives only topical treatment, and assess the efficacy of a combination of more than one modality for more improvement of cellulite.

## 5. Conclusions

In conclusion, this study showed that the effectiveness of ESWT was superior to MLD for the treatment of cellulite after liposuction as there was more reduction in the grade of cellulite in the ESWT group than the MLD group. Further studies are still required to assess the effect of ESWT and MLD on depression and quality of life after liposuction.

## Figures and Tables

**Figure 1:** The flowchart of the study.

**Figure 2:** Mean skinfold caliper before and after treatment of group A and B ^*∗∗*^: nonsignificant difference before treatment between group A and group B; ^*∗*^: significant difference after treatment between group A and group B.

**Figure 3:** Median values of the cellulite grading scale before and after treatment of group A and B ^*∗∗*^: nonsignificant difference before treatment between group A and group B; ^*∗*^: significant difference after treatment between group A and group B.

**Table 1:** Baseline characteristics.

Parameters	Group A, *n* = 15	Group B, *n* = 15	MD	*t* value	*p* value
Age (years)	36.06 ± 6.09	35.66 ± 4.95	0.4	0.19	0.84
Weight (kg)	93.13 ± 4.6	94 ± 3.89	−0.87	−0.55	0.58
Height (cm)	166.13 ± 2.66	165.6 ± 2.77	0.53	0.53	0.59
BMI (kg/m^2^)	33.76 ± 1.93	34.31 ± 2.01	−0.55	-0.76	0.45

Data are presented as mean ± standard deviation; significance is at *p* < 0.05; MD: mean difference.

**Table 2:** Mean skinfold caliper before and after treatment of group A and B.

Skinfold caliper (cm)	Group A, *n* = 15	Group B, *n* = 15	MD (95% CI)	*t* value	*p* value
Before treatment	8.36 ± 0.25	8.32 ± 0.21	0.04 (−0.12: 0.22)	0.54	0.59
After treatment	6.32 ± 0.17	7.04 ± 0.27	−0.72 (−0.89: −0.55)	−8.71	0.001
MD (95% CI)	2.04 (1.94: 2.15)	1.28 (1.1: 1.44)			
% of change	24.4	15.38			
*t* value	41.23	16.25			
*p* value	0.001	0.001			

Data are presented as mean ± standard deviation; significance is at *p* < 0.05; MD: mean difference; CI: confidence interval.

**Table 3:** Median values of cellulite grading scale before and after treatment of group A and B.

Cellulite grading scale	Group A *n* = 15	Group B *n* = 15	*U* value	*p* value
Before treatment	3 (3,3)	3 (3,3)	112.5	1.000
After treatment	1 (1,1)	2 (2,2)	40.5	0.001
*Z* value	3.49	3.62		
*p* value	0.001	0.001		

Data are presented as median (interquartile range); significance is at *p* < 0.05; *U* value: Mann–Whitney test value; *Z* value: Wilcoxon signed ranks test value.

## Data Availability

The authors declare that all relevant data supporting the findings of this study are available within the article.
